This article has been retracted.

# Hyperspectral Image Analysis of Colon Tissue and Deep Learning for Characterization of Health care

**DOI:** 10.1155/2022/8670534

**Published:** 2022-05-31

**Authors:** Ammar Akram Abdulrazzaq, Sana Sulaiman Hamid, Asaad T. Al-Douri, A. A. Hamad Mohamad, D. Selvi, Abdelrahman Mohamed Ibrahim

**Affiliations:** ^1^Department of Medical Laboratory Techniques, Al-maarif University College, Ramadi, Al-Anbar, Iraq; ^2^Al-Farahidi University, Communication Technical Engineering, Baghdad, Iraq; ^3^Department of Dental Industry, College of Medical Technology, Al-Kitab University, Kirkuk, Iraq; ^4^Department of Medical Laboratory Techniques, Dijlah University College, Baghdad 10021, Iraq; ^5^The University of Mashreq, Research Center, Baghdad, Iraq; ^6^Department of Physics, Jayaraj Annapackiam College for Women Periyakulam, Theni, Tamil Nadu, India; ^7^Accounting and Financial Management School of Management Studies, University of Khartoum, Khartoum, Sudan

## Abstract

Colon cancer is a disease characterized by the unusual and uncontrolled development of cells that are found in the large intestine. If the tumour extends to the lower part of the colon (rectum), the cancer may be colorectal. Medical imaging is the denomination of methods used to create visual representations of the human body for clinical analysis, such as diagnosing, monitoring, and treating medical conditions. In this research, a computational proposal is presented to aid the diagnosis of colon cancer, which consists of using hyperspectral images obtained from slides with biopsy samples of colon tissue in paraffin, characterizing pixels so that, afterwards, imaging techniques can be applied. Using computer graphics augmenting conventional histological deep learning architecture, it can classify pixels in hyperspectral images as cancerous, inflammatory, or healthy. It is possible to find connections between histochemical characteristics and the absorbance of tissue under various conditions using infrared photons at various frequencies in hyperspectral imaging (HSI). Deep learning techniques were used to construct and implement a predictor to detect anomalies, as well as to develop a computer interface to assist pathologists in the diagnosis of colon cancer. An infrared absorbance spectrum of each of the pixels used in the developed classifier resulted in an accuracy level of 94% for these three classes.

## 1. Introduction

Colon cancer is a condition characterized by the abnormal and uncontrolled growth of cells that are present in the large intestine, which is the source of the disease. If the tumour has spread to the lower region of the colon (rectum), it is possible that the cancer is colorectal in nature [1]. Colon cancer is a disease characterized by the unusual and uncontrolled development of cells that are found in the large intestine. If the tumour extends to the lower part of the colon (rectum), the cancer may be colorectal [1]. Adenomatous polyps, which grow on the intestine's inner walls and are usually benign, are the origin of the majority of colon cancers. Hematoxylin and eosin (H&E) staining is used in the majority of colon cancer examinations, as is the case with most cancer diagnoses [2].

Machine learning is a branch of computer science that has been extensively used in pre-diagnosis research [3]. The development of algorithms that can learn from their mistakes and predict future events is quite appealing. Rather than just following preprogrammed instructions, these algorithms build a model from input samples to make predictions or judgments. Machine learning has many subareas, such as artificial neural networks (ANNs), convolutional neural networks (CNNs), and ANN with deep learning architecture (or deep neural networks) [4]. The first is a set of computational models inspired by the nervous system that can learn and recognize patterns [5].

Many approaches have been developed to analyse HSI. Despite this variability, the use of HSI spatial information for tumour categorization is limited. Manni et al. [6] reviewed HSI analysis methods based on their classification approach. They are (a) preprocessing methods and (b) deep learning approaches (deep learning, DL). Methods for HSI analysis based on preprocessing procedures were adapted from traditional data analysis techniques. Initially, data modification and spectral band selection were utilized to solve HSI's high dimensionality. In this context, PCA and PLS approaches are commonly employed to extract spectral features [7] and support vector machines (SVMs) for spectral classification [8]. Later, recognizing the importance of spatial information in HSI classification, new spectra-spatial approaches were suggested, incorporating the dimensions *x*, *y*, and z. Spatial-spectral classification approaches improve spectral classification performance [9]. The wavelet transform (WT) has been widely employed in examining nonlinear features and kernel-based approaches (KM), such as kernel PCA and discriminant analysis in the Fisher core [10]. Manual approaches for HSI classification are still widely utilized in tumour diagnosis [11].

Deep learning has recently enhanced HSI categorization [12]. Tasnim et al. [13] created a five-layer CNN with basic CNN elements in the input layer. L'Heureux et al. [14] used HSI to diagnose thyroid cancer, while Dariya et al. [15] used HSI to diagnose colon cancer. It was trained on 50 patient samples of excised squamous cell carcinoma, thyroid cancer, and normal head and neck tissue. This work investigates the use of hyperspectral infrared images for pattern recognition and tissue anomaly identification. Each pixel requires a spectrum of hundreds or thousands of different frequencies. ANNs with deep learning architecture are efficient and effective ways to manage enormous datasets. An application can learn about a hyperspectral image's attributes and differences from previous classification records used to train a classifier. The use of ANN algorithms with deep learning architecture was chosen since they have been used widely and have produced some of the greatest results [16]. ANN with deep learning architecture thus stands out among the most widely used artificial intelligence methodologies because of its robustness and result quality. ANN with deep learning architecture seems promising for this purpose. The use of infrared spectra to identify aberrant colon tissue sections in biopsy samples will be explored, implemented, and assessed. The idea was to test whether hyperspectral images might identify aberrant tissue patches.

Spatial and Brightness Discrete Image (*x*,*y*). Assume that each row and column represents a single picture point. While the pixel is the smallest visual unit in two dimensions (*x* and *y*), it is closely followed by the voxel (*x*, *y*, and *z*). Each pixel in a digital image has spatial coordinates and numerical values. Each pixel in a grayscale image creates a two-dimensional data matrix. Images in red, green, and blue (RGB) (Figure 1) are constructed as a three-dimensional data matrix.

A spectral image is one that reproduces an object based on its wavelength. This type of imaging provides geographical and chemical information about the sample. Imaging uses a digital camera to capture spatial data, while spectroscopy uses a spectrometer to capture spectrum data. However, before editing hyperspectral images, they must be transformed into a data matrix. In a two-dimensional matrix, each pixel is a sample of intensity values (or frequencies), which are organized in lines according to the given order. Applications such as MATLAB make this possible. Basic and quick image segmentation algorithm is developed for the detection of inflammatory and malignant tumours in colon biopsy samples using infrared spectra. It is recommended for instances where identifying and extracting an object from a picture take a long time. This last phase used analytical cross-validation because the original experiment used a lot more data I achieved the following: similarity, segmentation, and edge detection and this is sufficient to prove the validity of the analysis.

Otsu Method: the Otsu approach maximizes the variance between picture classes, or the separation between object and image backdrop. Otsu is an object-oriented method. Otsu is a great solution for general real-time computer vision applications. Its sequential implementation sets a global threshold. The idea is to cycle through all possible edge values in an image, aiming for the one that minimizes the image's intraclass variance. This value separates foreground and background and assigns a color to each class. Equation (1) calculates the intraclass variance for a possible threshold *t*.

(1) $$\begin{array}{c} \sigma_{w}^{2}=w_{b}\sigma_{b}^{2}+w_{f}\sigma_{f}^{2}, \end{array}$$

where *w* is the weight for each class. This measure corresponds to the probability that a pixel has to belong to class *b* (background) or *f* (foreground).

## 2. Methodology

Current histological colon biopsy evaluations include tissue collection, colonoscopy, and pathologist analysis of the H&E picture. The time to diagnose depends on both the quality of the material and the professional's skill. Several studies propose optimizing this process in histological tests using technologies such as hyperspectral imaging and ANNs. There was no research on using hyperspectral imaging with RNA technology and deep learning architecture to characterize colon tissues in three classifications (cancer, inflamed, and healthy).

Hyperspectral imaging was thought to identify anomalies embedded in its pixels' spectrum and give the assisting in the diagnosis of colon cancer utilizing RNAs with deep learning architecture to assess pixels in hyperspectral pictures generated from slides with biopsy samples of colon tissue in paraffin but now was to identify inflammatory and malignant tumors in colon biopsy samples using infrared spectra. The application's goal is to supplement conventional histological examinations with a pre-diagnosis computer visual tool that helps develop more trustworthy and accurate diagnoses. The proposal also claims that hyperspectral scans may distinguish cancerous, inflammatory, and healthy tissue regions based on their pixel spectrum. Proposing the method proof requires various stages in the produced modules. Thus, the system used in the proposed experiment is composed of five modules, as follows:

- ROI Database Generator—system that automatically assembles the database that was used in the classifier training module, containing only the digital ROIs (and their respective 1626 hyperspectral frequencies) previously defined manually by the pathologist. The system automatically generates—in a single file—all ROIs from a database of hyperspectral images categorized in the CIS classification.
- Optimization and Cross-Validation—manually defining the best hyperparameters for an ANN with a deep learning architecture can be an expensive job. In order for the classifier training module to be executed more precisely, in this second step, it was proposed to implement a system that automatically selects the best hyperparameters from a native Keras resource: the best_params attribute of the GridSearchCV function. Once the best hyperparameters are defined, it is extremely important to validate the ANN with a deep learning architecture using different fractions of the ROI bank through an authenticator system that uses the cross-validation methodology [17].
- Classifier Training—after all the steps for generating the ROI bank and optimizing and validating the best RNA hyperparameters with a deep learning architecture, this implementation generates the file containing the weights and the final training that will be used in the production tooling.
- Production Tooling—the implementation allows loading a hyperspectral image of colon cancer biopsy at the input, enabling the classification of each of its pixels according to the CIS classification trained in the classify training module, generating a new digital image at the output colorized containing the pre-diagnosis result.
- Web Interface PAIH–friendly Web interface, easy to distribute, and that allows the pathologist and researchers to select and pre-diagnose hyperspectral images in a visual, quick, and simple way.

Figure 2 shows the operating process of the proposed application and the dependency between the developed modules, where

- It is the hyperspectral image file in its standard format (FSM)
- The file is then opened in the MATLAB application for metadata analysis
- The FSM file is converted and exported to CSV format
- Base (directory) of hyperspectral data in CSV format
- ROI bank generator module
- ROI bank, also in CSV format
- Classifier training module
- JSON file containing the structure of the ANN
- Production tooling module
- Application Web interfaces
- Visual pre-diagnosis result
- Parts that constitute the PAIH Web interface

### 2.1. Test Environment

To minimize the time of the experimentation phase of this research, two different test environments were used. The first is a conventional computer, intended for lighter processing tasks, such as the ROI bank generator, the production tooling, and the PAIH Web interface [16]. The second is a dedicated server, used in tasks that required more time and processing consumption, such as optimization and cross-validation and classifier training. The dedicated server belongs to the department of computing and mathematics (DCM) in our university. In both test environments, the same programs and libraries were installed, allowing all developed modules to be executed correctly in any environment. The algorithms of all modules were written using the Python programming language in its version 3.7.0. The Google TensorFlow 2.0 Machine Learning Library and the Keras 2.4 RNA API complete the basic test environment requirements for this research. Other supplementary technologies complemented the structure of the developed modules and will be specified in their respective subsections.

#### 2.1.1. Image Base

Both hyperspectral pictures of colon tissue and digital photographs stained with H&E were employed in this study. The pictures were taken from the open-source library. First, the photographs were created in FSM format and divided into three groups: 9 photographs identified as malignant, 9 as inflamed, and 9 as healthy. The input of the deep learning ANN classifier in matrix format is as follows: pixels in rows and frequencies in columns of the entity forming a hyperspectral image. The H&E digital images (Figure 3) help identify each hyperspectral image. The pathologist used the H&E pictures to label the pixels and mark the ROIs. Finally, the PAIH Web interface used these photographs to identify tests. This work's main output is hyperspectral image files. So, the first stage of the investigation was to learn how to read and alter these files. The images were created by an extractor utilizing MATLAB to extract data per pixel from these photographs. Because this is an unusual file type, the first step was to convert it to CSV. Results and discussions will explain why this conversion occurred [13].

### 2.2. ROI Bank Generator

When opening a hyperspectral image in FSM format in the MATLAB application, the system presents some entities that have, in addition to information about the pixels of the hyperspectral image, other important information about the file, such as the number of existing frequencies. This stage of the work aimed to understand the composition of these entities.

The main entities allocated in the metadata of a hyperspectral image are as follows:

- wn—the frequencies (total of 1626) referring to the wave number range (750–4000 cm^−1^).
- dy—the vertical pixel resolution of the hyperspectral image. In the example of Figure 4, 241 pixels are shown.
- dx—the horizontal pixel resolution of the hyperspectral image. In the example of Figure 4, 193 pixels are shown.
- R—the matrix containing the number of image pixels (dy multiplied by dx) by the number of frequencies.

The main entity, *R*, effectively retains the hyperspectral image's pixels and their 1626 frequencies. This entity's structure can be seen in MATLAB. The value corresponding to the matrix column in the *r* entity in the wn entity is checked to find the pixel absorbance value at the frequency corresponding to the wave number (1 to 1626). Other methods include converting numbers to cm1 using the equation: 750 + (2 ^*∗*^ matrix column r) - 2, where the result is 750 + 2 ^*∗*^ 1026 = 2800 cm^1^. According to Silva (2013), to view an image in one of the 1626 accessible frequencies, a column (frequency) must be converted to a new data matrix with width and height equal to the metadata's dy and dx entities. An algorithm in the ROI bank generator application does this automatically, but it can also be done with MATLAB's imshow (*m*(*x*,*y*,*z*)) function, where imshow displays 2D images, *m* is a hyperspectral image matrix, *x* is the number of horizontal pixels to display, *y* is the number of vertical pixels to display, and *z* is the hyperspectral frequency of the *z*-axis.  Figure 5 simulates the conversion.

The pathologist can then manually demarcate the detected locations with signs of malignancy, inflammation, or healthy tissue. The pathologist's free manual demarcations (Figure 5(c)) do not have the same number of pixels. So, beginning from the middle region of each manual demarcation, an uniform digital size of 50 × 50 pixels was created for all ROIs (Figure 5(d)), visually guaranteeing that each ROI, afterwards delimited in the hyperspectral picture, was placed within the pathologist's H&E image. As a result, all 27 ROIs have the same pixel resolution.

In generating the ROI base, used to train the ANN classifier with deep learning architecture, it was necessary to group the resolution information and coordinates of all 27 ROIs—specified with 50 × 50 pixels—in each image and store them in a database (Table 1) so that the module could generate the ROI base automatically from all the hyperspectral images in the image base. The ImageJ 6 program was used to locate the coordinates of the ROI.

### 2.3. Training and Optimization of the Network

The ROI base defined the ANN architecture for deep learning, but creating a hyperparameter architecture for each application remains difficult. Epochs, activation functions, and optimizers are hyperparameters. Manually testing several architectures takes time and effort. We optimize two scikit-learn machine learning hyperparameters. Without scikit-param learn's grid argument, a dictionary of hyperparameters must be provided. Apart from analysing each model (parameter set) in the dictionary, the cross-validation logo defines the result of two enhanced hyperparameters [16]. This study contains numerous parameter tests. Only the best after or tuning will be shown. Cross-validation is widely used in statistics and machine learning to avoid overfitting. We used it to define two hyperparameters and test the ROI foundation. The holdout method is the most frequent for ANNs. The dice is used for RNA training and testing. The base plot used for training should not exceed 70% of the total data volume. The remaining 30% is used to evaluate model accuracy. A contemporary attorney was utilized as a starting reference. This last phase used an analytical cross-validation because the original experiment used a lot more data. K-fold cross-validation: this method divides the dice into K equal-sized groups (called folds). The process is repeated K times, providing K test error estimates for each K group. According to James et al., the classifier's average performance in K tests is 5-10 pa. A potassium blood test measures the amount of potassium in the blood. To improve the ANN's accuracy, multiple testing is justified. In most cases, K-fold cross-validation with *K* = 5 or 10 is employed to quantify the test error and variance (used in this experiment). After constructing ROIs, we used deep learning and K-fold cross-validation to train a classifier [9, 12]. The ANN classifier used in this study can diagnose hyperspectral images of colon cancer. Determining how to save RNA training data was critical since deep learning processing RNA can take hours or days. The Keras supports saving the final ANN model with deep learning architecture as a JSON file. The research was named nn strusture.json in Figure 2(h). The Keras allows a second non-HDF58 file. Along with the model, they are saved in *n* weights.h5. Finally, the production tooling module will load these two files and run the classification method.

### 2.4. Production Equipment

Production tooling is the core of the proposed system in this project. This module loads or classifies RNA using deep learning architecture (JSON file generated in the classifier training module), allowing classification of pixels in a hyperspectral image and pre-diagnosis of colon cancer biopsy examination. First, production tooling loads two files: nn strusture.json and nn weights.h. One of the challenges of this undertaking was separating the two paraffin areas. In the classifier training module, the classifier is limited to thirty regions matching tissues [4]. Non-biopsy tissue might create unwanted non-pre-diagnostic results, leading to false positives. The next procedure is to separate the hyperspectral image of the biopsy from the paraffin image. So, three DIP approaches are used: OTSU threshold, expansion, and erosion. In this case, a hyperspectral frequency was used to base a binary mask on. According to experts from the Photo Biophysics Laboratory, we utilized a frequency corresponding to a wave number equal to 1600 cm^−1^ to define the binary mask in this phase. Finally, using a binary mask, the object (fabric) is removed from the image background (paraffin) and brightness, peaks, and values are calibrated using dilation and erosion methods to limit fabric material loss.

The entire method Figure 6 employed the Python OpenCV9 package [12]. A library contains dozens of thresholding routines to help developers. Once the binary mask is created, the system compares the pixel coordinates of the hyperspectral image with the binary mask where, if the mask value is 0, the classifier ignores this pixel and production tooling defines its color as black. Two pixels are classified in this stage for pre-diagnosis. Other 3 matrices are generated: one for cancerous pixels (mC), one for inflamed pixels (mI), and one for healthy pixels (mH) (mS). Production tooling transmits all hyperspectral frequencies to the classifier or pixel for examination. The pixel is carcinogenic, and thus, production tooling just colors it red in the mC matrix. If the candidate pixel is inflamed, its mi matrix coordinate is green. Finally, bright pixels are blue in the mS matrix.

At the end of the process, the system generates a digital image in portable network graphics (PNG) format, in which each channel or RGB channel matrix corresponds to the colorization carried out by the RNA with the deep learning architecture (mC, mI, and mS), delivering no end to colorization two pixels per category. The production tooling also presents the user with the % age of pixels classified in each category. These stages constitute the pre-diagnosis of the system and will be detailed in results and discussions.

### 2.5. PAIH Web Interface

At the last stage of the project, the objective is the development of the layer of user interface (UI) that enables a simple interaction with the system. The UI operates as the frontend of production tooling, which, from a more technical point of view, deals with the backend litter of the system. Together with both layers, they complement the PAIH application.

The PAIH was developed with the objective of making it simpler for the user to interact with an RNA engine with deep learning architecture, proposed in this research. The frontend was programmed using the Web-enabled libraries (flask) of the Python programming language, as well as a set of development patterns and practices that facilitate code structure and reuse, such as design patterns [18] and other Internet technologies, such as HTML5, CSS, JSON, JavaScript, and AJAX. The initial interface, or PAIH, allows two types of possible actors to use the tool, either a researcher or a pathologist. Depending on the selected profile, the information presented does not subject the system to access alterations. In general, users with a researcher level have unrestricted access to the system files, and users with a pathologist level can only manipulate hyperspectral images in CSV, view digital H&E images, and perform pre-diagnoses. The limitation of access occurs because there is no need for pathologist users to have access, for example, to the FSM files, once they are used only in research activities, mainly aiming at contributions in future work. As its access by third parties violates the application rules, the application automatically recognizes and organizes directories and subdirectories containing a set of system-compatible files, such as hyperspectral images (FSM), digital images (PNG or TIFF), and CSV files. These directories are located on a server, making PAIH a repository of colon tissue biopsy tests in the cloud. To select a hyperspectral image in the selection box, the user can press the pre-diagnosis [10] button so that the production tooling engine is activated and the pre-diagnosis is processed. At the end of the process, the system exhibits H&E image, a hyperspectral frequency corresponding to a wave number equal to 1600 cm^−1^, or a colorized pre-diagnosis result in a PNG image with a CIS classification and a % age of RNA success with deep learning architecture. It is possible to notice that the hyperspectral image and the H&E image [15] do not have the same resolution, ratio, and rotation and are still clearer than the highlight circle in Figure 7. This is an important point to be mentioned, so that there are no doubts regarding the authenticity of the pre-diagnosis performed by PAIH. This detail, despite being common and not presenting any problems in the RNA classification process with deep learning architecture, is present in all the images used in this research.

## 3. Results and Discussions

### 3.1. Basis of ROIs

In the end, 27 ROIs were extracted (one of each available hyperspectral image), being 9 carcinogenic, 9 inflamed, and 9 healthy. Each ROI has a dimension of 50 × 50 pixels (total of 2500 pixels) and each pixel has 1626 frequencies to be analysed by the RNA with deep learning architecture. In sum, the pixels are the instances to be analysed and the frequencies are the attributes of each instance. The total number of pixels based on ROIs was 67500 pixels, with a disk volume totaling approximately 1.2 GB. As a way of validating the algorithm, the application will generate in a directory a ROI in PNG format (Figure 8). Despite the proven efficiency of the algorithm in executing the ROI cut, we believe it is important to carry out this concept test to minimize the probability of errors in the process. All the pixels are organized on the basis of ROIs following the same scheme explained in Figure 5, where the lines represent pixels and the columns represent frequencies. It is important to highlight the reason for the conversion of the FSM file to CSV in this project. As mentioned, because it is an atypical file format, the first stage consisted of the conversion of the FSM format to another more popular one, which could be used.

All the resources of the two packages NumPy and Pandas of the Python programming language are enjoyed. Also, it was defined as CSV extension, a very common file format, easy to manipulate, and compatible with various Python resources. The conversation was carried out using the export function of the MATLAB application, which made it possible to identify important information (metadata) about two image files.

### 3.2. Tuning

Based on the nonmanual API of Keras and the related works described in Section 2 (state of the art), three different configurations have been tested using the GridSearchCV function. Each set of hyperparameters was referred to here as a scenario. At the end of the process, the GridSearchCV function returns the best hyperparameter to be used on the basis of ANN training with deep learning architecture, from the best_params attribute. The tuning process carried out was executed in the test environment of the dedicated server and the entire process lasted approximately 20 days and 6 hours. Foram tested the following hyperparameters:

- Units: it refers to the number of neurons used in hidden litters.
- Batch_size: it is the number of batch samples used in one iteration.
- Activation: it defines the best activation function.
- Optimizer: it is an algorithm used to maximize the performance of the network in gradient descent.
- Epochs: it is the process cycle of the proposed scenario in architecture, in which it is repeated until some stop criterion is reached, normally the fact of changing weights will become very small.

It is important to highlight that there are works, which propose new methods and discuss the predefinition of hyperparameters for tuning to optimize the performance of an ANN. In this work, we opted for the use of the GridSearchCV function, but without leaving aside the importance of optimizing two hyperparameters, since the objective of this research phase is still part of the principle of validating the purpose of classifying two pixels. Also, other optimization models could be tested in future jobs.

### 3.3. Assessment

The cross-validation K-fold presented excellent results of accuracy in the three proposed scenarios in the tuning process. As shown in the graph of Figure 9, despite having a great difference in accuracy between the 1st scene and the other two, the difference in accuracy between the 2nd and 3rd scenes was practically null, when it exceeded 1000 processing times, oscillating in decimal values around 94%. Scenario 1 remained with an accuracy of around 80%, even arriving a 3000 epochs.

With this, let us keep as a choice Scenario 3, which despite having or doubling two values of the batch_size hypermeter and three times more times than Scenario 2, it did not present a significant difference in processing time, reaching an accuracy of 94.4%, no case, 0.2% more efficient than the Scenario 2, which showed 94.2% accuracy.

### 3.4. Pre-Diagnosis Tool

The first test executed in the PAIH tool was the pre-diagnosis of the 27 hyper-respective images that were used in the extraction of the ROIs for the construction of the classifier. The objective of this stage was to analyse whether the predominant class coincided (or did not) with the previous classification indicated by the pathologist.  Figure 10 presents the results in the following order: (i) image ID: it identifies the selected file, where the first initial of the file corresponds to its class (CIS); (ii) class: it corresponds to the previous classification indicated by the pathologist (CIS); and (iii) accuracy of the RNA pre-diagnosis in each class (cancer, inflamed, or healthy): it is defined as the % age of pixels correctly classified in relation to class (highlighted in green).

All the 27 images obtained predominance in relation to the diagnosis previously made by the pathologist, with the majority giving an accuracy between 80% and 99%, indicating the efficiency of the developed classifier. Still, analysing each case, in the class of files with initials in C (carcinogenic), the highest accuracy was from the C11 file (Figure 11(a)), achieving 99.9% success and the lowest accuracy was from the C21 file (Figure 11)., achieving 71.2% correct. Mostly two files of this class obtained values above 88% correct, being the class better classified. In relation to the files with initials in I (inflamed), the highest accuracy was obtained in file I1 (Figure 11(c)), reaching 98.2% of success, and the lowest accuracy was obtained in the file I5 (Figure 11(d)), reaching 66.4% success. In this class, most of the two files also obtained values above 80% correct. Finally, in a class of files with initials in S (healthy), the highest accuracy was obtained in the S12 file (Figure 11(e)), reaching 99.5% correct, and the lowest in the S2 file (Figure 11(f)), reaching 54.2% success rate, being the lowest ranking among all the classes. In this class, most of the two files also obtained accuracy values above 80%.

Finally, there is no pre-diagnosis validation process for the production tooling of the PAIH application, so we will not participate in the final pre-diagnosis test in the 27 photographs used to construct the base of ROIs and trained no classifier. The results matched a pathologist's manual diagnosis. As seen in Figure 10(g), the color red dominates. The ANN with deep Learning architecture also accurately diagnoses the hyperspectral image, with 92.6% of the tissue area identified as cancer, 7.4% as inflamed (green), and 0% as healthy (blue). Figure 11(h) shows a green color predominance, with 71.9% of the tissue classified as inflammation, 3% as cancer, and 25.1% as healthy. Finally, Figure 11(i) is largely blue, with 81.3% healthy fabric, 17.7% cancer, and 1% inflammation. Inflammatory tissue is common in malignant sites. Figure 3 shows 7.4% of inflammatory tissues. Despite their small size, the red dots in Figure 3 may indicate a classifier error. Since each pixel must be classified, 27 ROIs are a respectable number, but for a production system, additional new examples based on ROIs would be required to refine or train the classifier. The classifier's result will be the larger or better set of tests, and the error estimate will be the larger or more exact set of tests. In certain circumstances, homogenization algorithms can help. Similarly, the CIS categorization of a hyperspectral image could be separated into homogenous zones based on a color characteristic and then evaluated individually or together. Finally, considering the test conditions, the computing cost was also noteworthy. Pre-diagnosis of production tooling in a conventional computer system has proven to be quite efficient, taking roughly 45 seconds for each exam. This time was nearly the same on a dedicated server. Despite the categorization process's complexity, the system proved to be quick enough in a production context. Nonetheless, in all testing, the categorization process used a lot of RAM. No ordinary computer (16 GB RAM) or classification method used 3–5% of RAM per pre-diagnosis (480–800 MB), indicating no dedicated server. In a Web environment, where tens or hundreds of tests might be run simultaneously, we believe that a more thorough investigation of this usage in a production setting is required.

## 4. Conclusions

The aim of this study was to identify inflammatory and malignant tumours in colon biopsy samples using infrared spectra. Hyperspectral imaging was thought to identify anomalies embedded in its pixels' spectrum. It can classify pixels in hyperspectral images as cancerous, inflammatory, or healthy. This pre-diagnosis of colon cancer is based on two classifier tests and two studies.

Our findings reveal that RNA structural changes caused by Web applications (PATH) can facilitate the direct binding of m6A-modified RNAs to low-complexity sites in RNA binding proteins.

The tool's design allows future research on hyperspectral pre-diagnosis of problems to be added into its engine.

- Two PAIH resources can be revalued from the generation of new RNA structures and hyperparameters utilizing deep learning architecture, simply by importing a new JSON file for the hardware.
- This allows researchers to quickly generate batch pre-diagnosis data.
- The Web module works on any device with a standard Web browser because the system does not need add-ons or cookies.
- Various users may have varying levels of access, allowing data manipulation.

One of the app's flaws is converting two FSM files to CSV. The dependency on the program can cause issues. In addition, training two pixels from a ROI base takes a long time. On a dedicated server, the training will last roughly 48 hours. Using new input images as passive artefacts for future training may necessitate precise scheduling between application uses and training period environment. Advanced settings and methods can be assessed once additional data and circumstances are understood.

Only a pathologist's interpretation can give true meaning to the data, generating the examination's diagnosis. A second pathologist's perspective may increase precision and reduce subjectivity [19].

### 4.1. Future Work

As proposals for future work, we can mention the following:

- ROIs are read and built from two FSM files of hyperspectral pictures straight to speed up the procedure.
- Co-registration techniques are used to align the H&E image with the hyperspectral image.
- Homogenization algorithms are used to reduce false positives in two-pixel classification and make the digital image, content, or pre-diagnosis result more aesthetically appealing for two-user interpretation.
- Evaluating alternatives further, while the results in Figure 8 show a modest oscillation between scenarios 2 and 3, we believe that fresh scenario recommendations may produce different results. 94% accuracy was enough to allow us to advance in all phases of the investigation.
- The PAIH tool's visual resources are improved to allow pathologists to digitally demarcate new ROIs in hyperspectral images for ANN classifier integration with deep learning architecture.

## Figures and Tables

**Figure 1:** Image data matrix: (a) in gray scales and (b) in RGB.

**Figure 2:** Scheme of functioning and dependence of the processes developed in the research.

**Figure 3:** Set of 27 H&E images used to identify hyperspectral images in the image base and to demarcate ROIs by the pathologist.

**Figure 4:** Composition of the main entities that are part of the structure of a hyperspectral image file in FSM format.

**Figure 5:** Simulation of how the rearrangement of a hyperspectral frequency is performed to generate a 2D image: (a) FSM hyperspectral image; (b) matrix rearranged according to dx and dy resolutions and (c) converted 2D image; (c) simulation of the demarcation performed manually by the pathologist in the H&E image; and (d) ROI (red square) digitally defined from manual demarcation, with a dimension of 50 × 50 pixels in the hyperspectral image.

**Figure 6:** Paraffin removal process and classification of two pixels.

**Figure 7:** (a) Hyperspectral image at a frequency corresponding to a wave number equal to 1600 cm^−1^; (b) H&E image. Both face the same examination, as shown or highlighted circle, but they have different spatial characteristics.

**Figure 8:** Hyperspectral image and its ROI, both at a frequency corresponding to a wave number equal to 1600 cm^−1^.

**Figure 9:** Comparison of accuracy between the proposed scenarios for ANN with deep learning architecture.

**Figure 10:** Results of the pre-diagnosis test on the images used in the extraction of ROIs for the construction of the classifier.

**Figure 11:** Ratio of two highest and lowest results by class and results of the pre-diagnosis performed by production tooling: (g) image C18 with a predominance of cancer (red); (h) image I1 with a predominance of inflammation (green); (i) S10 image with a predominance of healthy tissues. All coincide with the previous classification indicated by the pathologist.

**Table 1:** Database of the ROI database generator module containing information on hyperspectral images (from left to right): image name, horizontal resolution, vertical resolution, ROI coordinate on the *x*-axis, and ROI coordinate on the *y*-axis and image class (CIS).

1	Image	*x*	*y*	coord_*x*	coord_*y*	coord_id↓
2	c4	193	241	102	99	c↓
3	c6	104	253	118	12	c↓
4	i1	204	253	144	104	i↓
5	i2	551	283	63	277	i↓
6	s12	272	128	37	199	s↓
7	s15	182	232	155	124	s↓

## Data Availability

The data underlying the results presented in the study are available within the manuscript.
